This article has been retracted.

# Discovering Gene Signature Shared by Prostate Cancer and Neurodegenerative Diseases Based on the Bioinformatics Approach

**DOI:** 10.1155/2022/8430485

**Published:** 2022-06-28

**Authors:** Qiang Su, Bin Dai, Hanjian Zhang, Shengqiang Zhang

**Affiliations:** ^1^Clinical Laboratory Medicine, Beijing Shijitan Hospital, Capital Medical University, Beijing 100038, China; ^2^Neurosurgery Department, Beijing Shijitan Hospital, Capital Medical University, Beijing 100038, China; ^3^Medical Affairs Department, Reckitt Benckiser (China) Holding Co., Ltd., Beijing 100020, China

## Abstract

**Background:**

Prostate cancer (PCa) is one of the highest frequent malignant tumors with very complicated pathogenesis. Genes of neurodegenerative diseases can influence tumor progression. But its role in the progression of PCa remains unclear. The purpose of the present academic work was to identify significant genes with poor outcome and their underlying mechanism.

**Methods:**

The GSE70768, GSE88808, and GSE134051 datasets were downloaded to screen the differentially expressed genes (DEGs). The DEG screening criteria were as follows: *P* < 0.05 and differential fold change |logFC| ≥ 1. The common DEGs (co-DEGs) of the three datasets were obtained by the Robust Rank Aggregation (RRA) method. Gene Ontology (GO) function annotation and Kyoto Encyclopedia of Genes and Genome (KEGG) pathway analysis were performed using R software. Protein-protein interaction (PPI) network analysis was performed for co-DEGs using STRING to screen critical genes. Differential expression and prognosis of key genes were analyzed by the online tool Gene Expression Profiling Interactive Analysis 2 (GEPIA2). The intersection gene between key genes and neurodegenerative genes was identified by constructing a Venn diagram.

**Results:**

A total of 263 co-DEGs were identified from the three datasets. GO analysis showed that co-DEGs were mainly involved in muscle contraction and blood circulation regulation. The top ten key genes were ACTG2, APOE, F5, CALD1, MYH11, MYL9, MYLK, TPM1, TPM2, and CALM1. GEPIA2 analysis showed that APOE, MYH11, and MYLK differ dramatically between tumor and normal tissues. These key genes are related to disease-free survival (DFS) in PCa. APOE was the intersection gene between key genes and Alzheimer-related genes.

**Conclusion:**

The neurodegenerative gene APOE may be a potential prognostic and diagnostic biomarker for PCa.

## 1. Introduction

Although the prevalence of neurodegenerative diseases and tumors increases with age, there is much evidence of inverse comorbidity of these two conditions [1, 2]. A strong correlation has been found between PCa and Alzheimer's disease (AD) [3]. However, the genetic risk shared by the two diseases remains unclear.

Global cancer statistics reveal that the incidence of PCa is the most common malignancy in males with 14.8% of the cases, sorting it the second highest in incidence and fifth highest in mortality [4]. Currently, the gold standard for clinical diagnosis of PCa is a prostate needle biopsy. However, the prostate needle biopsy leads to a higher incidence of hematuria, pain, and infection. Prostate-specific antigen (PSA) has several limitations as an early detection biomarker for PCa [5]. Benign prostatic hyperplasia (BPH) and prostatitis also give rise to elevated serum PSA levels [6]. Furthermore, PSA screening sometimes leads to overdiagnosis or overtreatment of PCa [7]. Therefore, it is very important to find new biomarkers of PCa with higher specificity and to explore the clinical significance of these biomarkers.

Recently, more and more microarrays and next-generation sequencing (NGS) technologies have been used to explore new biomarkers and therapeutic targets for PCa [8]. Nonetheless, the data volume of a single dataset is relatively small and the results are not reliable. In addition, it is difficult to process and analyze data in multidatasets. To solve the problem, the RRA technique was used, which is suitable for analyzing multiple gene datasets and can screen out more robust key genes [9, 10].

This study performed RRA analysis using three microarray datasets from the GEO database to identify co-DEGs between PCa and normal tissues. Bioinformatics analysis was performed to find key genes. Expression and survival analysis of key genes in The Cancer Genome Atlas (TCGA) database were performed using the online tool GEPIA2 to verify their prognostic and diagnostic value for PCa. We used Venn diagrams to find common risk genes for both diseases.

## 2. Materials and Methods

### 2.1. Data Sources

We selected eligible datasets using the following criteria: (a) the dataset must include both normal prostate tissues and PCa tissues and (b) each group had a sample size greater than 30. Three datasets (GSE70768, GSE88808, and GSE134051) were screened from the GEO database (http://www.ncbi.nlm. http://nih.gov/geo). The GSE70768 dataset was derived from the GPL10558 platform and contained 74 normal prostate tissues and 112 PCa tissues. The GSE88808 dataset was derived from the GPL22571 platform and contained 49 normal prostate tissues and 49 PCa tissues. The GSE134051 dataset was derived from the GPL26898 platform and contained 36 normal prostate tissues and 216 PCa tissues. The expression data were normalized by the “normalize between arrays” function in the R package “limma.”

### 2.2. Screening of Co-DEGs

The DEGs in each dataset were filtered using the R package “limma” (https://bioconductor.org/packages/limma). Adjusted *P* values (adjust. *P*) < 0.05 and ‖log fold change (FC)‖ > 1 were set as the cutoff values to screen DEG. The RRA method-based R package “RobustRankAggreg” was utilized for the integrated analysis of the DEGs. Co-DEGs were obtained by the integrated upregulated and downregulated DEG lists. The log FCs of co-DEGs were presented as averages of three GSE datasets.

### 2.3. GO and KEGG Enrichment Analysis

GO functional and KEGG pathway enrichment analysis was implemented via the “clusterProfiler” package (https://bioconductor.org/packages/clusterProfiler). GO was classified into three aspects of biology: Biological Process (BP), Molecular Function (MF), and Cellular Component (CC).

### 2.4. Construction of the PPI Network

Interaction PPI networks of co-DEGs were analyzed by the online database STRING (https://string-db.org/) with high confidence score > 0.7. Visualizing PPI networks hid points that are not associated with any other gene. The top ten connectivity co-DEGs were defined as key genes.

### 2.5. Prognostic Analysis

PCa patients were divided into low- and high-expression groups according to the median expression value of key genes. The GEPIA2 database (http://gepia2.cancer-pku.cn/) was an online database for prognostic analysis of tumor samples from TCGA [11].

### 2.6. Venn Analyses

Expression and survival analysis of key genes were performed using GEPIA2. The neurodegenerative genes were obtained by literature [1]. Venn graphs were delineated to identify common biomarkers in PCa and neurodegenerative diseases by the Venn tool (http://bioinformatics.psb.ugent.be/webtools/Venn/).

### 2.7. Statistical Analysis

Statistical analysis was performed with R software (version 3.6.3). Continuous variables were compared between two groups via the Wilcoxon rank-sum test. Kaplan-Meier survival curve analysis and log-rank test were used for survival analysis. *P* < 0.05 was considered statistically significant.

## 3. Results

### 3.1. Data Integration and Co-DEG Identification

In the GSE70768 dataset, 709 DEGs were identified and are shown in Figure 1(a). In the GSE88808 dataset, 1640 DEGs were identified and are shown in Figure 1(b). In the GSE134051 dataset, 926 DEGs were identified and are shown in Figure 1(c). A total of 263 co-DEGs were excavated from three datasets by RRA analysis (117 upregulated and 146 downregulated). The top 20 up- and downregulated co-DEGs of each dataset are displayed in Figure 1(d).

### 3.2. GO and KEGG Enrichment Analysis of Co-DEGs

GO function analysis using the R package “clusterProfiler” and the top 10 results of GO terms are displayed in Figure 2(a). Co-DEGs were mainly enriched in the muscle system process for BP, collagen-containing extracellular matrix for CC, and calmodulin binding for MF. KEGG analysis revealed that co-DEGs were mostly allocated in six pathways. Two major KEGG pathways were focus adhesion and vascular smooth muscle contraction (Figure 2(b)). The relationship between co-DEGs and pathways is shown in Figure 2(c).

### 3.3. Construction of the Core PPI Network

The core PPI network was constructed using the STRING online database, as shown in Figure 3(a). The node degree represents the connectivity degree between co-DEGs. The key genes from the top 10 node degrees in the PPI network are as follows: ACTG2, APOE, F5, CALD1, MYH11, MYL9, MYLK, TPM1, TPM2, and CALM1 (Figure 3(b)). The neurodegenerative genes were composed of 19 genes from the study of Gargini et al. [1] and are shown in Table 1.

### 3.4. Prognostic Significance of Key Genes

GEPIA2 was utilized to identify the differential expression and prognosis of key genes in TCGA database. Nine key genes showed significantly different expressions between normal and cancer tissues (Figure 4(a)). In addition, three genes (APOE, MYH11, and MYLK) were found to be associated with disease-free survival (DFS) (Figure 4(b)). To intuitively and effectively learn which differential genes are commonly owned in different groups, we use the Venn diagram to obtain the overlapped genes. The results showed that one hub gene (APOE) was shared by the key genes and neurodegenerative genes (Figure 4(c)).

## 4. Discussion

The incidence of PCa has been rising globally [12]. In China, PCa accounts for 8.16% of all male tumors, ranking sixth, and the mortality rate is 13.61%, ranking seventh [13]. Multiple risk factors are related to the transformation, progression, and death of PCa, such as race, family history, diet, smoking, and genomic alterations [14]. Although most localized PCa has a good prognosis after surgical treatment, its high incidence and varying prognosis present challenges for patients and physicians, both from the risk of undertreatment as well as overtreatment [15]. Also, patients with PCa after radical surgery have a high recurrence rate (30%) [16]. Currently, the treatment protocol for PCa depends on clinical and pathological prognostic biomarkers such as PSA, T staging, and Gleason score [17]. The National Comprehensive Cancer Network (NCCN) guidelines can stratify the risk of the patient and provide further diagnosis and treatment recommendations. However, the clinicopathological features of the guidelines do not fully and reliably reflect the intrinsic biology of the tumor and often misclassify the aggressiveness of the tumor [18]. For example, while needle biopsies of the prostate are the gold standard for diagnosing PCa in men, there is still a risk of false negatives [19]. TPSA lacks specificity for PCa and may lead to unnecessary biopsies [20]. The Gleason score is based on a pathologist's assessment of the cancer tissue [21] and has too much variability among different pathologists [22]. Imaging is difficult to detect early malignancy in the prostate, as well as for long-term follow-up to assess survival probability. Magnetic resonance imaging (MRI) and other imaging biomarkers cannot improve survival rates, and 12% of cancer cases were missed by multiparameter MRI [23, 24]. The above methods are difficult to be used as the main methods for large-scale early screening of PCa. In addition, many novel markers cannot be used in the clinic due to the lack of normalized diagnostic protocols [19, 25].

The genetic risk of PCa is associated with aggressiveness and poor prognosis, which suggests an urgent need to increase genetic screening [26]. Genetic factors accounted for 57% of the etiology of PCa. Men with BRCA1 or BRCA2 germline mutations have an approximately 4-fold and 9-fold higher risk of PCa, respectively, than men without the mutations. Other low-risk genetic variants have also been identified, and genomic characteristics and structural variations in PCa have been associated with cancer metastasis [27]. Therefore, translating the results of basic scientific research into biomarkers of clinical value for diagnosis and prognosis is crucial for precision medicine in PCa [28]. In particular, screening and early diagnosis of PCa have yet to become common in China.

In this study, datasets GSE70768, GSE88808, and GSE134051 were analyzed by the RRA method and 263 co-DEGs were found. Then, GO functional annotation shows that co-DEGs are mainly involved in BP: muscle contraction and blood circulation regulation, CC: collagenous extracellular matrix and contractile fiber and myofibrils, and MF: calmodulin binding, cytoskeleton composition, and muscle composition. These results suggest that co-DEGs are related to the proliferation and migration of PCa. KEGG pathway analysis showed that these co-DEGs were mainly enriched in the following six pathways: focal adhesion, vascular smooth muscle contraction, oxytocin signaling pathway, pancreatic secretion, salivation secretion, and drug metabolism-cytochrome P450. In the focal adhesion pathway, focal adhesion kinase (FAK) plays an important role in the development and progression of PCa. The mechanism may be that tyrosine kinase signals through integrin-activated FAK to promote cell proliferation, metastasis, and angiogenesis [29]. In vascular smooth muscle contraction pathways, smooth muscle contraction of the prostate and the lower urinary tract has been implicated as a cause of urinary disease and related to higher morbidity and mortality [30]. Oxytocin signaling pathway, pancreatic secretion pathway, salivary secretion pathway, and drug metabolism-cytochrome P450 pathway are rarely seen in the field of PCa.

In the present study, a PPI network was constructed and revealed ten key genes. GEPIA2 analysis showed that the expression levels of APOE, MYH11, and MYLK were related to DFS in PCa. Some studies have shown that MYLK was a new marker for predicting the biochemical recurrence of PCa [31]. It has also been confirmed that circRNA-MYLK is an oncogene of PCa, and its mechanism is that the upregulation of circRNA-MYLK promotes the development of PCa by targeting miR-29a [32]. Some studies have shown that decreased MYH11 expression level in lung cancer patients is related to poor prognosis, mainly involved in biological processes such as “muscle contraction,” “contraction of the fiber part,” “actin cytoskeleton,” and “adhesion and connection” [33]. MYH11 is rarely studied in the development of PCa and can be a prognostic biomarker and therapeutic target for PCa.

As a gene associated with AD, APOE has higher expression in PCa than in normal tissue. The APOE E4 allele is a risk factor for AD and might be a risk factor for prostate cancer as well [34]. This may be related to vascular lesions, which can lead to the progression of prostate cancer and neurodegenerative disease [35]. This is consistent with the conclusion found by our enrichment analysis of co-DEGs: the mechanism of PCa progression is related to vascular smooth muscle contraction pathway and blood circulation regulation function. It may help choose the optimal treatment for PCa and AD.

## 5. Conclusions

In conclusion, the present study improved the understanding of the molecular mechanism of PCa development by bioinformatics analysis and identified key genes related to PCa progression. The key gene APOE in this study may be a potential diagnostic and prognostic biomarker for PCa and neurodegenerative diseases.

## Figures and Tables

**Figure 1:** Volcano plots and heatmap reflecting significant DEGs in GSE134051, GSE70768, and GSE88808. (a–c) Volcano plots reflect significant DEGs in GSE134051, GSE70768, and GSE88808, respectively. (d) Heatmap of each expression microarray. Red: upregulated differential genes; green: downregulated genes; black: no significant differential genes.

**Figure 2:** GO and KEGG analysis of co-DEGs. (a) Top 10 enriched GO terms of co-DEGs. (b) KEGG enrichment analysis results of the co-DEGs. (c) The plot presents the relationship between co-DEGs and six pathways. GO: Gene Ontology; KEGG: Kyoto Encyclopedia of Genes and Genome; co-DEGs: common differentially expressed genes.

**Figure 3:** PPI network analysis of co-DEGs. (a) PPI network of co-DEGs. (b) The bar graph indicates the node degree of the top 25 co-DEGs. PPI: protein-protein interaction networks; co-DEGs: common differentially expressed genes.

**Figure 4:** Differential expression and DFS analysis of key genes in prostate cancer patients. (a) Boxplot of top 10 co-DEG expressions in TCGA dataset. (b) DFS analysis of top 10 co-DEGs using GEPIA2. (c) Venn diagram of key and neurodegenerative genes. ^∗^*P* < 0.05. num: number; T: prostate tumor group; N: normal group; DFS: disease-free survival.

**Table 1:** Genes of neurodegenerative diseases.

	Neurodegenerative-related genes
Alzheimer	APP, Tau/MAPT, PSEN1, PSEN2, APOE, and GSK3B
Parkinson	GBA, LRRK2, PARK2 (PRKN), PARK7, PINK1, SNCA, and UCHL1
Amyotrophic lateral sclerosis	C9orf72, TARDBP, SOD1, FUS, UBQLN2, and HNRNPA2B1

## Data Availability

The data and materials used to support the findings of this study are available from the corresponding author upon request.

## Abbreviations

APOE: Apolipoprotein E
ACTG2: Actin gamma 2
F5: Coagulation factor V
CALD1: Caldesmon 1
MYH11: Myosin heavy chain 11
MYL9: Myosin light chain 9
MYLK: Myosin light chain kinase
TPM1: Tropomyosin 1
TPM2: Tropomyosin 2
CALM1: Calmodulin 1.
